RETRACTED

# Effect of Comprehensive Nursing on the Recovery of Gastrointestinal Function in Patients Undergoing Abdominal Operation

**DOI:** 10.1155/2022/1179321

**Published:** 2022-08-21

**Authors:** Lanlan Xiang, Wei Liu, Yuanyuan Jin

**Affiliations:** ^1^Pediatric Surgery Department of Gastrointestinal Surgery, The First People's Hospital, Jingmen, Hubei Province, China; ^2^Department of Gastroenterology, The First People's Hospital, Jingmen, Hubei Province, China

## Abstract

**Objective:**

The objective is to explore the effect of comprehensive nursing on the recovery of gastrointestinal function in patients undergoing an abdominal operation.

**Methods:**

Sixty patients undergoing abdominal surgery in our hospital from January 2019 to April 2021 were enrolled. The patients were arbitrarily assigned into control group and research group. The former group received routine nursing and the latter group received comprehensive nursing. Nursing satisfaction, gastrointestinal function, POMS-SF score, nutrition risk score, incidence of adverse reactions, and quality of life scores were compared.

**Results:**

The nursing satisfaction of the research group was higher than that of the control group, and the difference between the groups was statistically significant (*P* < 0.05). In terms of gastrointestinal function, the anal exhaust time eating time defecation time and bowel sound recovery time in the research group were significantly lower than those in the control group, and the difference between the groups was statistically significant (*P* < 0.05). In terms of POMS-SF score, the scores of tension–anxiety, depression–depression, fatigue–dullness, anger–hostility, and confusion–confusion in the research group were lower than those in the control group, while the energy-vitality score was higher than that in the control group, and the difference between the groups was statistically significant (*P* < 0.05). There was no significant difference in nutritional risk score among patients before nursing (*P* > 0.05); after nursing, the nutritional risk score decreased. Compared between the two groups, the nutritional risk score of the research group was lower when compared to the control group at 3 days, 5 days, and 7 days after nursing, and the difference between the groups was statistically significant (*P* < 0.05). In terms of the incidence of adverse reactions, the incidence of adverse reactions such as incision effusion, incision infection, incision dehiscence, and anastomotic leakage in the research group was lower when compared to the control group, and the difference between the groups was statistically significant (*P* < 0.05). Regarding quality of life scores, before nursing, there exhibited no significant difference of patients (*P* > 0.05); after nursing, the quality of life scores of patients decreased. Compared with the two groups, the physical function, psychological function, social function, and healthy self-cognition scores of the research group were all lower compared to the control group, and the difference between the groups was statistically significant (*P* < 0.05).

RETRACTED

**Conclusion:**

Abdominal surgery patients received comprehensive care, which improved their mental health, reduced anxiety and depression levels, relieved fatigue and dullness, improved energy and vitality, and enhanced their overall mood. Meanwhile, it can also promote the recovery of gastrointestinal function in patients and reduce the incidence of adverse reactions.

## 1. Introduction

After the diagnosis of patients undergoing abdominal surgery, there are often a variety of bad emotions that affect the patient's eating, resulting in insufficient nutritional intake and low spirits; the operation will cause harm to the body, which is bound to consume a lot of nutrition, thus affecting the recovery of gastrointestinal function [1]. Gastroparesis is one of the common complications of abdominal surgery, especially after radical gastrectomy and pancreaticoduodenectomy [1]. Most of it occurs 1 to 2 days after the open diet or when the patient transitions from a liquid diet to a semi-fluid diet. The main symptoms are fullness or upper abdominal compression, no severe abdominal pain, vomiting a small amount to a large amount of gastric juice, containing bile; the symptoms can be significantly relieved after vomiting. Once it occurs after the operation, it often lasts for weeks, months, or even longer, so it is extremely difficult for clinical diagnosis and treatment. Due to different diagnostic criteria, the incidence of gastroparesis reported in some literature is 0.3% to 10% [2]. The incidence of gastroparesis after gastrectomy can be as high as 4.7% [3]. The etiology of gastroparesis after abdominal surgery is not yet clear, which may be related to the following factors: (1) whether there is gastric outflow tract obstruction before surgery: generally, patients with gastric outflow tract obstruction before surgery are more likely to develop postoperative gastric outflow tract obstruction than those without obstruction. more chance of gastroparesis; (2) whether there is an underlying disease that affects gastrointestinal motility: such as diabetes, hypothyroidism, scleroderma, etc.; (3) the way of reconstructing the digestive tract after gastrectomy: patients who underwent Billroth II anastomosis were more the incidence of gastroparesis is higher; and (4) the scope and degree of intraoperative lymph node dissection: the wider and more thorough the lymph node dissection, the more chance of gastroparesis. Basic studies have found that the possible mechanisms of gastroparesis are as follows [4, 5]. The main results are as follows: (1) surgical trauma itself activates the sympathetic nervous system and enhances the inhibitory activity of gastrointestinal sympathetic nerve in vivo. The activated sympathetic nerve fibers can not only inhibit the excited neurons of the gastrointestinal plexus but also inhibit gastric motility by directly binding the catecholamines released from the sympathetic nerve endings to the *α* and *β* receptors on the membrane of gastric smooth muscle cells, then inhibit the contraction of smooth muscle cells; (2) if the stomach is operated on, it will damage the vagus nerve or destroy the structural integrity of the stomach, resulting in an imbalance of gastric emptying; and (3) the secretion, metabolism, and regulation of gastrointestinal hormones are also affected to a certain extent [4].

RETRACTED

With the progress of modern surgical theory, the concept of rapid rehabilitation surgery has gradually formed and changed the traditional model of gastrointestinal surgery since the beginning of this century, overturning many practices that are accustomed to, but have no evidence-based medicine [5]. Among them, the abandonment of nasogastric tube before and after the operation and the encouragement of early diet after operation attract people's attention. From past experience, surgeons generally take it for granted that nasogastric tubes are used in gastrointestinal surgery, in addition to maintaining gastric emptying during anesthesia and reducing the incidence of aspiration during operation. It can also promote the recovery of postoperative gastrointestinal function and reduce the occurrence of nausea, vomiting, abdominal distension, and pulmonary complications. However, current clinical evidence shows that patients who do not routinely use nasogastric tubes recover intestinal function earlier and have a lower incidence of pneumonia [6–8]. The concept of rapid rehabilitation surgery also requires that patients be given a small amount of water and an open liquid diet on the day after operation, and gradually increase the amount and transition to a normal diet within a relatively short period of time after operation, and stop intravenous rehydration as soon as possible [9]. However, there is a contradiction between the renewal of modern surgical ideas and clinical reality. On the one hand, the number of elderly patients and severe patients after major surgery increased, the recovery of gastrointestinal function in these groups was slow, and the possibility of gastroparesis was remarkably higher compared to normal patients. Aspiration can cause reflux of gastric contents, which often leads to aspiration pneumonia and can be life-threatening [10]. On the other hand, rapid rehabilitation surgery requires early eating without a gastrointestinal decompression tube from the point of view of reducing perioperative trauma and stress, promoting early rehabilitation, shortening hospitalization days, and saving hospitalization costs. Therefore, how to identify the high-risk population of gastroparesis after abdominal surgery and take necessary measures to reduce the risk of reflux aspiration has deeper clinical significance than before. Comprehensive nursing intervention can be traced back to the middle of the 19th century; the United States took the lead in putting forward case management (CM), that is, managing patients as a whole. After a century of development, the term integrated management was formally formed in the middle of the 20th century, from which comprehensive nursing was developed and integrated with the thinking mode of the nursing procedure [11]. Comprehensive nursing is a new way of clinical nursing intervention, which is a perfect combination of nursing measures implemented by nurses in the process of holistic and comprehensive nursing for patients, in order to achieve an auxiliary method for the treatment of diseases [12]. Comprehensive nursing intervention needs to use multi-disciplinary knowledge to deal with the problems in clinical practice, through case assessment, planning, implementation, feedback, and adjustment, take appropriate nursing measures to meet the needs of patients. At present, the comprehensive nursing intervention has been widely adopted in various clinical fields. Some scholars have pointed out that comprehensive nursing measures such as cognitive intervention, progressive muscle relaxation training (PMR intervention), and group psychological intervention are adopted to observe the patients' mood, coping style, and quality of life before and within one month after receiving a comprehensive nursing intervention. The results indicated that comprehensive nursing intervention improved the mood of lung cancer patients undergoing chemotherapy, made patients adopt a positive coping style and enhanced their quality of life [13]. Based on this, the purpose of this study is to explore the effect of comprehensive nursing on the recovery of gastrointestinal function in patients undergoing abdominal surgery.

RETRACTED

## 2. Patients and Methods

### 2.1. Normal Information

Sixty patients undergoing abdominal surgery in our hospital from January 2019 to April 2021 were enrolled. The patients were randomly divided into control group and research group. The former group received routine nursing and the latter group received comprehensive nursing. There were 18 males and 12 females in the control group and 17 males and 13 females in the research group with an average age of (45.31 ± 3.55) years (1974 years) and (45.75 ± 3.53) years (17 males and 13 females). There exhibited no statistical significance in the general data. This study was permitted by the Medical Ethics Association of our hospital, and all patients noticed informed consent. This study is a double-blind trial.

Selection criteria: meet (1) 18 years ≤ age ≤80 years old, ASA I ∼ II, 18 kg/*m*2 ≤ BMI ≤30 kg/m2; (2) no previous cardiovascular and respiratory diseases; (3) no chest wall trauma or chest deformities; and (4) the expected duration of the operation is more than 3 hours.

Exclusion criteria: meet (1) ASA grade ≥3; (2) severe hypertension and heart disease; (3) moderate or severe restrictive or obstructive pulmonary disease; and (4) anemia (hemoglobin is lower than 100 g/L).

### 2.2. Treatment Methods

The control group received routine nursing intervention in the department, issued disease guidance manuals to patients on the day of admission, evaluated admission, patiently carried out health education to patients, and explained to patients matters needing attention in disease-related self-management. Individual nursing guidance was given, and health education was the main way of education.

The research group received comprehensive care with the following specific measures:

1. A comprehensive nursing team was established, consisting of 2 senior medical oncology deputy chief physicians, 1 nutritionist, 1 psychological counseling and therapist, and 4 ward nursing responsible nurses (including head nurses and senior responsible nurses), a total of 8 people composition. Establish an intervention information file, uniformly register the enrolled patients, record the chemotherapy cycle and the date of each hospitalization and discharge, and collect survey data in a planned way; establish a WeChat group for patients in the intervention group, and push nutrition education information to patients irregularly after discharge. Comprehensive care team members review and answer patient nutritional and psychological questions every night.
2. Formulate comprehensive nursing intervention measures: use “comprehensive nursing”, “adjuvant chemotherapy”, “nutrition risk”, “comprehensive nursing”, “adjuvant chemotherapy”, and “nutritional risk” as search words to search China knowledge Network, Wanfang, PubMed, Medline, and other databases, read the relevant literature, refer to the implementation methods of comprehensive nursing, and review and discuss the literature by the members of the group, and implement it after being reviewed by the experts in the hospital to ensure the scientific nature and feasibility of comprehensive nursing intervention measures. The final formulation of comprehensive nursing intervention measures includes: (1) nutritional assessment and education; (2) nutritional supplement intervention; and (3) psychological intervention.
3. Implementation of comprehensive nursing intervention measures:

Nutrition assessment and education: (1) after the patient was admitted to the hospital for the first time, the nurse in charge of the research group was responsible for receiving the patient, helping the patient understand the bed attending doctor, familiar with the ward environment, and creating a good bed environment. A good atmosphere for medical treatment lays a good foundation for further research. (2) Nutrition assessment: when admitted to the hospital for the first time, the responsible nurses used the dietary retrospective method to evaluate the nutritional status of patients and their families. The assessment included dietary rules, type and quantity of food intake, dietary nutritional requirements, and the presence or absence of partial eating, food fear, and food allergy, and asked patients about the main ways of intake of nutritional knowledge and assessed whether there were nutritional misunderstandings, etc. to fully understand the nutritional status of patients, so that dietitians can make personalized nutrition education plans for patients according to the results of the assessment; (3) Nutrition education: according to the individualized nutrition education plan, the responsible nurses adopted IIFAR information nursing method to carry out nutrition knowledge education to patients for 15–20 minutes each time [14]. IIFAR scheme: initial check: check the information the patient needs and choose the best time for the patient to receive the information. Information exchange conveys information and communicates to patients through a variety of forms. Through face-to-face conversation, we can distribute brochures to formulate nutritional meals according to dietary guidelines, watch nutrition promotion videos, organize patient education meetings, explain the contents of the bulletin board to patients, and carry out education according to their needs. WeChat can also promote nutrition science knowledge and other channels to ensure that patients receive information effectively. Final accuracy check: ensure the accuracy and validity of the information conveyed. Patients were asked about their learning experience at the end of each education and after re-admission, and patients were encouraged to briefly retell the learning content, deepen memory, and correct wrong cognition in time to prevent cognitive deviation, and reactions were adopted to evaluate whether patients mastered communication knowledge and whether their nutritional status had improved. Regular follow-up was conducted after discharge, and patients were asked about food intake, weight changes, and gastrointestinal discomfort reactions, and specific dietary guidance was given.

RETRACTED

Nutritional supplement intervention: the daily food intake and times of patients in the intervention group were supervised and recorded by responsible nurses, and the eating situation and discomfort reaction of patients were observed. According to the results of the first PG-SGA assessment and the diet of the patients within one week after the first chemotherapy, the comprehensive nursing intervention group discussed the formulation of a specific nutritional intervention plan, which was constantly revised with the nutritional status of the patients. Patients in each chemotherapy cycle: according to the five-step model of nutritional intervention, oral nutritional supplement (ONS) is the first choice. Patients who cannot eat by mouth or those with severe gastrointestinal reactions can be supported by the placement of an enteral nutrition tube or peripheral intravenous nutrition, or the combination of parenteral and enteral nutrition. The prescription of parenteral nutrition and parenteral nutrition was jointly formulated by the research team, and the responsible nurses gave corresponding nursing measures, including parenteral nutrition nursing and enteral nutrition nursing.

Psychological intervention: (1) supportive psychotherapy: including mental health education and psychological emotion regulation. Responsible for nurses and head nurses to conduct psychological interviews with the families of newly admitted patients before chemotherapy, to understand the basic situation of patients, including family background, interests, understanding of the disease, and expectations of treatment, and to formulate a detailed treatment plan. According to the actual situation of patients to develop psychological counseling program for patients, specific methods remove unreasonable cognition and correctly understand the disease: medical staff uses their own professional knowledge to provide patients with professional guidance on the main treatment, adverse reactions, nursing, prognosis, and other aspects of the disease, so that patients have a more in-depth understanding of the occurrence and development of the disease, medical effects, and other aspects, so as to improve their cognitive level of disease treatment and their own situation. Help them understand the law of disease development and avoid negative psychological effects and negative emotions due to a lack of understanding of the disease; (2) guide the correct psychological cognition in the face of the disease: use accurate, distinct, kind, kind and positive language to communicate with the patients, guide the patients to face the disease correctly and reverse the traditional concept formed for a long time. Gradually eliminate the patients' fear of the disease itself and treatment, face the disease with an optimistic attitude, so as to achieve the goal of treating the disease and promoting physical and mental health; (3) instruct patients to carry out effective emotional regulation: teach patients to identify their own negative emotions, timely dredge, manage or establish the ability to seek help actively, carry out self-regulation and nursing in time, and effectively correct emotional problems. Enhance the ability of self-awareness and self-correction, and get rid of negative emotional problems such as pessimism and disappointment as soon as possible. Relaxation therapy: relaxation therapy refers to training and learning, so that patients can consciously control their physical and mental activities, relax tension, achieve a state of peace of mind, physical and mental harmony, reduce the level of arousal, and adjust the function of the body from tension. From the second day of hospitalization, the psychological counseling therapist guided the patients to train according to the relaxation training procedure once a day in the afternoon. The specific methods are: (1) arrange a clean and quiet room with soft light, take a comfortable lying position and close your eyes slightly; (2) tell the patient to take a deep breath. Keep the rhythm natural and steady and focus on breathing; (3) according to certain instructions, patients are guided to tighten a certain muscle group first, and then relax, which can be carried out in the order from top to bottom, so as to relieve tension and anxiety; (4) after all parts of the body are relaxed, let this comfort be maintained for 3–5 minutes; (3) individualized psychological intervention: (1) in-depth communication: through in-depth communication between counseling therapists and patients and main caregivers, to understand the patient's personality and emotional characteristics, family-social situation, the process of seeking medical treatment and the cognition of disease and treatment. Fully understand the true thoughts of the patients and encourage them to express their doubts; (2) psychological counseling: give counseling, explanation, and comfort to patients with specific questions, fully combine “speech therapy” with “chemotherapy”, and cooperate with necessary psychotherapy according to the situation, such as music therapy, suggestion therapy. Patients with a high matching degree and remarkable therapeutic effect can also be enrolled according to the situation to carry out collective psychological intervention with the patients in the intervention group, through common communication and learning, to explore good coping behavior, and to carry out psychological solutions and persuasion. To help patients eliminate tension and anxiety and improve their determination to overcome the disease; (3) family and social support: explain to the family members the important role of family support and help in the treatment and rehabilitation of patients, encourage them to actively cooperate with treatment and nursing, pay attention to the psychological changes of the main caregivers, and dredge patients with greater psychological stress. Provide positive emotional support for patients and reduce their psychological burden.

RETRACTED

### 2.3. Observation Index

#### 2.3.1. Satisfaction

After consulting the literature and experts' discussion, we designed patients' follow-up satisfaction, a total of 10 items, and recorded patients' satisfaction with follow-up management mode, health education, medical and nursing service, and appointment registration process [12]. It is assigned into four dimensions: very satisfied, satisfied, general, and dissatisfied. Satisfaction rate = very satisfaction rate + satisfaction rate + general rate.

### 2.4. Gastrointestinal Function

#### 2.4.1. Profile of Mood States. Short Form (POMS-SF)

The reliability of the Chinese simplified POMS questionnaire ranges from 0.62 to 0.82, with an average r-0.71, and the reliability is high. Chinese scholar Wang Jianping confirmed that the discrimination, reliability, and validity of POMS-SF in cancer patients met the requirements of psychometrics and were suitable for the detection of the emotional status of cancer patients in clinical practice [15]. POMS-SF consists of a subscale of six emotional situations: a positive scale: energy-vigor scale. The higher the score, the better the mood. The five subscales are negative scales: tension–anxiety (POMST), fatigue–retardation (POMSF), depression–depression–depression (POMSD), confusion–confusion (POMSC), and anger–hostility (AHPOM). The higher the score, the worse the mood. The total score (TMD) can be adopted as a separate indicator.

#### 2.4.2. Nutrition Risk Screening Table

Nutrition risk screening table nutritional risk screening 2002, NRS-2002NRS2002, is based on a systematic review of 128RCT and is a nutrition assessment tool issued by the European Society for Parenteral Nutrition (EPSPEN) in 2003. Kondrup analyzed the reliability of NRS2002, its Kappa value is 0.67, and its content validity is expounded on the basis of literature research, so as to ensure a good content validity [16]. The scale consists of three parts: disease severity, nutritional damage, and age score, and is divided into the sum of the above three scores, that is, 0–7 × NRS2002 score <3 indicates no nutritional risk, and NRS2002 score ≥3 indicates nutritional risk.

RETRACTED

#### 2.4.3. Incidence of Adverse Reactions

The incidences of adverse reactions such as incision effusion, incision infection, incision dehiscence, and anastomotic leakage were calculated.

#### 2.4.4. Quality of Life Scale

The quality of life scale consists of four subscales, including physical, psychological, social, and health self-awareness, with a total of 29 items [17]. The Cronbach's *α* coefficient of the scale is 0.79 to 0.91. The scale was scored by 1–5 grades. The lower the score, the higher the satisfaction.

### 2.5. Statistical Analysis

Using SPSS21.0 statistical software, before statistical analysis, the measurement data were examined by normal distribution and variance homogeneity analysis to meet the requirements of a normal distribution or approximate normal distribution, presented as $\bar{x}\pm s$, and repeated measurement data were analyzed by repeated measurement analysis of variance. *T* test was adopted to compare the two groups, *n* (%) was adopted as an example to represent the counting data, and *χ*2 test was adopted. *P* < 0.05 indicated that the difference between the groups was statistically significant.

## 3. Results

### 3.1. Comparison of Nursing Satisfaction

In terms of nursing satisfaction, the research group was very satisfied in 24 cases, satisfactory in 5 cases, and general in 1 case, with a satisfaction rate of 100.00%; In the control group, 14 cases were very satisfied, 10 cases were satisfied, 1 case was general, and 5 cases were dissatisfied. The satisfaction rate was 83.33%; The nursing satisfaction of the research group was higher compared to the control group, and the difference between the groups was statistically significant (*P* < 0.05). All the data results are indicated in Figure 1.

### 3.2. Comparison of Gastrointestinal Function

In terms of gastrointestinal function, the anal exhaust time eating time defecation time and bowel sound recovery time in the research group were significantly lower than those in the control group, and the difference between the groups was statistically significant (*P* < 0.05). All the data results are indicated in Table 1.

RETRACTED

### 3.3. POMS-SF Score Comparison

In terms of POMS-SF score, the scores of tension–anxiety, depression–depression, fatigue–dullness, anger–hostility, and confusion–confusion in the research group were lower than those in the control group, while the energy-vitality score was higher than that in the control group, and the difference between the groups was statistically significant (*P* < 0.05). All data results are indicated in Table 2.

### 3.4. Comparison of Nutritional Risk Scores

There was no significant difference in nutritional risk score before nursing (*P* > 0.05) but decreased after nursing. Compared with the two groups, the nutritional risk score of the research group was lower than that of the control group on the 3rd, 5th, and 7th day after nursing, and the difference between the groups was statistically significant (*P* < 0.05). All the data results are indicated in Table 3.

### 3.5. Comparison of the Incidence of Adverse Reactions

Regarding the incidence of adverse reactions, the incidence of adverse reactions such as incision effusion, incision infection, incision dehiscence, and anastomotic leakage in the research group was lower compared to the control group, and the difference between the groups was statistically significant (*P* < 0.05). All data results are indicated in Figure 2.

### 3.6. Quality of Life Score Comparison

There was no significant difference in the score of quality of life before nursing (*P* > 0.05) but decreased after nursing. The scores of physiological function, psychological function, social function, and health self-cognition in the research group were lower than those in the control group, and the difference between the groups was statistically significant (*P* < 0.05). All the data results are indicated in Table 4.

## 4. Discussion

Delayed gastric emptying due to gastrointestinal motility disorders after abdominal surgery is collectively referred to as functional gastric emptying disorder or gastroparesis [17]. Therefore, during the comprehensive treatment of patients undergoing abdominal surgery, we must pay attention to the nutritional status of patients, such as not taking timely measures to improve the nutritional level of patients, and the decline of immunity of patients under malnutrition; it will have a negative impact on the treatment effect and prognosis. Professor Shi Hanping proposed that nutrition education is the basic content of nutrition intervention and the first choice of nutrition therapy [18]. In the clinic, there are many nutritional misunderstandings in tumor patients, and the most common misunderstandings are taboos, thinking that supplementary nutrition will accelerate the growth of tumor cells. There are also more common misunderstandings, such as over-reliance on health products and superstitious vegetarian diet. The American Society for Parenteral and Enteral Nutrition (ASPEN) pointed out that reasonable nutritional intervention can effectively enhance the nutritional status of patients and remarkably promote their immunity [19]. Therefore, it is particularly important to eliminate bad cognition, spread scientific and healthy nutrition knowledge, provide reasonable and correct dietary nutrition advice for patients with nutritional needs, cooperate with effective nutritional intervention, and improve the nutritional status of patients. Comprehensive nursing intervention plays a positive role in delaying the loss of weight and nutritional index of patients undergoing abdominal surgery [19, 20]. Through reasonable and effective comprehensive nursing intervention for patients undergoing abdominal surgery, we can reduce the negative impact of chemotherapy on the body, reduce the decline of patients' nutritional levels, and play a positive role in maintaining postoperative nutritional level. In the study of scholars, in the multi-disciplinary nursing intervention for patients undergoing abdominal surgery, it was found that there exhibited no statistically significant change in the nutritional index grade of the patients in the intervention group after 21 days of observation, and there exhibited a statistically significant difference after follow-up observation for 1 month, which is consistent with the results of this study. It indicates that nutritional intervention needs a process, and with the extension of time, it can indicate the advantage of its effect on the nutritional status of patients undergoing abdominal surgery. In this study, due to the short observation period, the more far-reaching and positive effect of comprehensive nursing intervention on the nutritional status of tumor patients need to be extended to the whole chemotherapy cycle in the future. Studies by some scholars have proved that nutritional support has a positive effect on improving the nutritional status of patients undergoing chemotherapy and the treatment of patients after abdominal surgery, which is similar to the results of this study [20]. Patients undergoing abdominal surgery often have some self-reported symptoms, such as nausea and vomiting, anorexia, and abdominal distension. Comprehensive nursing increased the part of patients' self-evaluation, fully considered the eating situation and the symptoms affecting eating, and effectively made up for the deficiency of relying solely on objective indicators to judge the nutritional status of patients. Studies of the 10th National gastric *Cancer* Congress and the third Sunshine Great Wall *Cancer* Congress also show that nutritional support during chemotherapy for patients undergoing abdominal surgery can improve nutritional status, enhance immunity and reduce adverse reactions caused by chemotherapy, similar to the results of this study [21]. From this, it can be inferred that the integration of management and maintenance evaluation and education into comprehensive nursing intervention measures can effectively enhance the nutritional status of patients undergoing abdominal surgery.

RETRACTED

With the continuous progress of modern medicine, the mental health of patients has been paid more attention by the medical community [22]. WHO's new definition of health points out that patients should be treated as a whole, and the attention to diseases is not limited to the scope of somatic diseases, but also to the mental health of patients. We can notice the importance of social and psychological factors to human physical and mental health [23]. After learning about the condition, patients with abdominal surgery will suffer a certain psychological impact, resulting in negative, evasive, and depressive emotions, and many patients are difficult to get rid of their own negative emotions, which seriously affect their quality of life and confidence in treatment [24]. Clinical observation shows that patients undergoing abdominal surgery have large mood fluctuations before and after operation, which leads to a concentrated outbreak of negative emotion in a short time. A large number of studies have shown that patients undergoing abdominal surgery have higher scores of anger, anxiety, depression, and fear than normal people [25–27]. With the extension of the rehabilitation cycle, the expression of bad emotion is more obvious. Previous studies have indicated that the causes of adverse psychological status in patients undergoing abdominal surgery are usually as follows: (1) stress reaction caused by confirmed disease; (2) worry about side effects after operation [28]; and (3) economic burden and self-perceived burden [29]. The cost of surgical treatment brings a huge financial burden to the patient's family. Repeated hospitalization and chemotherapy cause the loss of family role, which makes the patient produce negative emotions that drag down the family and become a family burden. As a result, negative emotions such as self-remorse, helplessness, depression, guilt, and anxiety appear. Therefore, when the patient's body and mind are extremely fragile, they need more care, support, and understanding from the family. Spiritual assistance and life care from family members play a positive role in building up confidence in overcoming the disease and improving treatment tolerance; (4) the uncertainty of the therapeutic effect and outcome of the disease [30]. At this stage, it is not enough to cure all cancers, the fear of death threats will also stimulate people's strong desire for survival and psychological expectations of the effectiveness of treatment, coupled with frequent and uncertain tumor metastasis. Anxiety and depression occur in patients with recurrent or worsening conditions; and (5) the influence of the hospital physical environment and social environment [31]. Compared with the psychological comfort brought by the family, the unfamiliar hospital environment is easy to make patients nervous, fear, and other discomfort, repeated hospitalization makes patients have a conditioned reflex to the hospital environment, in addition, some medical staff cannot clearly feel the emotional changes of patients, impatience and kindness in the process of inquiring about the patient's condition or explaining matters needing attention may lead to negative psychological emotion. We can find that the causes of adverse psychological emotions in patients undergoing abdominal surgery are complex and need to be treated because of illness, and psychological intervention can get twice the result with half the effort if we give corresponding psychological intervention to the causes of the problems [32].

RETRACTED

To help patients improve poor nutritional status, get rid of negative emotional disorders, and maintain a good physical and mental state to receive disease treatment is a necessary nursing measure for patients undergoing abdominal surgery. This study shows that comprehensive nursing intervention can effectively reduce the decline of patients' nutritional levels, alleviate the degree of anxiety and depression, and promote the improvement of patients' overall mood. It is suggested that the comprehensive nursing intervention program should be further promoted in clinical work to improve the malnutrition and psychological state of patients with malignant tumors undergoing adjuvant chemotherapy. With the continuous development of nutrition, the nutrition furuncle treatment group (NST) appeared one after another and assumed the important responsibility of clinical nutrition knowledge dissemination and education. Due to the lack of understanding of the importance of NST, there are still few nutrition specialist nurses in our country. At present, the main clinical nutrition work is mainly undertaken by nutrition nurses [33]. However, in the actual work, the clinical nurses are closest to the patients and have more frequent contact. Training nutrition specialist nurses and setting up a comprehensive nursing team are more conducive to the implementation of the nutrition nursing plan. In the survey of patients undergoing abdominal surgery, it was found that 99.6% of patients had dietary misunderstandings, 93% of patients had not received formal nutrition education, and 70% of patients had doubts about how to eat scientifically [34]. The first two sources of nutrition knowledge for patients undergoing abdominal surgery are television (56.5%) and medical staff (54.4%), while the last two are magazines (25.5%) and dietitians (10.2%) [35, 36]. Medical staff and dietitians did not play their due role in nutritional treatment. Some data show that 76% of patients are not satisfied with clinical nutrition knowledge, 63% of patients want to receive nutrition knowledge education from nurses, and only 11% of nurses think that their nutrition knowledge reserve can meet the needs of patients [37, 38]. It can be noticed that clinical nurses are lack of professional nutrition knowledge. In the future talent echelon construction, we should pay attention to the training of specialist nurses and the establishment of a comprehensive nursing team. As people pay more attention to mental health, psychological intervention nursing, as a new nursing model, has been gradually integrated into clinical nursing work in recent years. A number of studies have indicated that it can play an important role in the treatment of diseases with negative emotions such as anxiety and depression, and can effectively improve the quality of life of tumor patients [39–41]. In view of the fact that at present, psychological support and psychological intervention are mostly completed by nurses and lack of professional training and guidance, the professional study and training of psychological nursing should be strengthened in the future in order to ensure the safety of patients and enhance the effect of an intervention. The same idea can be found in the study put forward by other scholars [42, 43]. They have applied new methods in the study, and the conclusions drawn can also give some support to this study. There are some limitations to this study. First, the sample size of this study is not large and it is a single-center study, so bias is inevitable. In future research, we will carry out multi-center, large-sample prospective studies, or more valuable conclusions can be drawn.

RETRACTED

In summary, patients undergoing abdominal surgery received comprehensive care, which enhanced their mental health, reduced the degree of anxiety and depression, relieved fatigue, dullness, energy, and vitality, and improved their overall mood. At the same time, it can also promote the recovery of gastrointestinal function and reduce the occurrence of adverse reactions.

## Figures and Tables

**Figure 1:** Comparison of nursing satisfaction between the two groups.

**Figure 2:** Comparison of the incidence of adverse reactions between the two groups.

**Table 1:** Comparison of gastrointestinal function between the two groups [$\bar{x}\pm s$,d].

Grouping	N	Anal exhaust time	Feeding time	Defecation time	Bowel sound recovery time
Control group	30	2.05 ± 0.22	2.36 ± 0.34	2.89 ± 0.21	2.05 ± 0.36
Research group	30	1.73 ± 0.12	1.95 ± 0.12	2.16 ± 0.21	1.65 ± 0.31
*t*		6.994	6.228	13.463	4.611
*P*		＜0.05	＜0.05	＜0.05	＜0.05

**Table 2:** Comparison of POMS-SF scores between the two groups [$\bar{x}\pm s$, points].

Groupating	*N*	Tension-anxiety	Depression-depression	Fatigue-retardation	Anger-hostility	Confusion-chaos	Energy-vigor
Control group	30	9.98 ± 1.44	8.93 ± 1.21	6.78 ± 1.21	5.79 ± 0.53	5.65 ± 1.21	4.31 ± 1.22
Research group	30	7.35 ± 1.21	7.45 ± 1.21	4.43 ± 0.31	4.41 ± 0.63	4.13 ± 0.31	6.42 ± 0.95
t		7.658	4.737	10.304	9.180	6.665	7.474
P		＜0.05	＜0.05	＜0.05	＜0.05	＜0.05	＜0.05

**Table 3:** Comparison of nutritional risk scores between the two groups [$\bar{x}\pm s$, points].

Grouping	N	Before nursing	After nursing 3 d	After nursing 5 d	After nursing 7 d
Control group	30	4.96 ± 0.53	3.84 ± 0.31	3.05 ± 0.31	2.95 ± 0.31
Research group	30	4.98 ± 0.51	3.01 ± 0.31	2.64 ± 0.12	2.56 ± 0.11
t		0.148	10.369	6.755	6.493
P		＞0.05	＜0.05	＜0.05	＜0.05

**Table 4:** Comparison of quality of life scores between the two groups [$\bar{x}\pm s$, points].

Grouping	N	Physiological function		Psychological function		Social function		Healthy self-cognition	
		Before nursing	After nursing	Before nursing	After nursing	Before nursing	After nursing	Before nursing	After nursing
Control group	30	15.57 ± 4.64	13.13 ± 2.33a	16.67 ± 3.53	14.34 ± 4.31a	18.76 ± 3.64	16.66 ± 2.66a	15.75 ± 3.53	13.55 ± 1.77a
Research group	30	15.53 ± 4.42	11.23 ± 2.55 b	16.96 ± 3.83	12.66 ± 1.12 b	18.77 ± 3.54	12.64 ± 3.67 b	15.66 ± 3.83	10.54 ± 2.63 b
t		0.034	3.012	0.304	2.066	0.010	4.857	0.094	5.200
P		＞0.05	＜0.05	＞0.05	＜0.05	＞0.05	＜0.05	＞0.05	＜0.05

*Note.* comparison before and after nursing in the control group, ^a^*P*＜0.05; Comparison before and after nursing in the research group, ^b^*P*＜0.05.

## Data Availability

The datasets used and analyzed during the current study are available from the corresponding author upon reasonable request.
